This article has been retracted.

# Mitochondrial-Associated Protein LRPPRC is Related With Poor Prognosis Potentially and Exerts as an Oncogene *Via* Maintaining Mitochondrial Function in Pancreatic Cancer

**DOI:** 10.3389/fgene.2021.817672

**Published:** 2022-02-14

**Authors:** Li Wang, Jun Luo, Yuchen Li, Yanrong Lu, Yi Zhang, Bole Tian, Ziyi Zhao, Qiong-ying Hu

**Affiliations:** ^1^ Department of Pancreatic Surgery, West China Hospital of Sichuan University, Chengdu, China; ^2^ School of Medicine, Chengdu Women’s and Children’s Central Hospital, University of Electronic Science and Technology of China, Chengdu, China; ^3^ College of Medical Technology, Chengdu University of Traditional Chinese Medicine, Chengdu, China; ^4^ Key Laboratory of Transplant Engineering and Immunology, West China Hospital of Sichuan University, Chengdu, China; ^5^ Department of Laboratory Medicine, Hospital of Chengdu University of Traditional Chinese Medicine, Chengdu, China

**Keywords:** LRPPRC, autophagy/mitophagy, pancreatic cancer, mitochondrial homeostasis, chemoresistance, reactive oxygen species (ROS)

## Abstract

**Background:** The mitochondrial-associated protein leucine-rich pentatricopeptide repeat-containing (LRPPRC) exerts multiple functions involved in physiological processes, including mitochondrial gene translation, cell cycle progression, and tumorigenesis. Previously, LRPPRC was reported to regulate mitophagy by interacting with Bcl-2 and Beclin-1 and thus modifying the activation of PI3KCIII and autophagy. Considering that LRPPRC was found to be negatively associated with survival rate, we hypothesize that LRPPRC may be involved in pancreatic cancer progression *via* its regulation of autophagy.

**Methods:** Real-time quantitative polymerase chain reaction was performed to detect the expression of LRPPRC in 90 paired pancreatic cancer and adjacent tissues and five pancreatic cancer cell lines. Mitochondrial reactive oxidative species level and function were measured. Mitophagy was measured by performing to detect LC3 levels.

**Results:** By performing a real-time quantitative polymerase chain reaction, the association of LRPPRC with the prognosis of pancreatic cancer was established, and pancreatic cancer tissues had significantly higher LRPPRC expression than adjacent tissues. LRPPRC was negatively associated with the overall survival rate. LRPPRC was also upregulated in pancreatic cancer cell lines. Knockdown of LRPPRC promoted reactive oxidative species accumulation, decreased mitochondrial membrane potential, promoted autophagy/mitophagy, and induced mitochondrial dysfunction. Subsequently, knockdown of LRPPRC inhibited malignant behaviors in PANC-1 cells, including proliferation, migration, invasion, tumor formation, and chemoresistance to gemcitabine. Finally, by inhibiting autophagy/mitophagy using 3-MA, the inhibitory effect of LRPPRC knockdown on proliferation was reversed.

**Conclusion:** Taken together, our results indicate that LRPPRC may act as an oncogene *via* maintaining mitochondrial homeostasis and could be used as a predictive marker for patient prognosis in pancreatic cancer.

## Introduction

Pancreatic cancer is one of the leading causes of cancer-related death and has a very low overall survival rate of approximately 5% and a median survival of less than 6 months (Siegel et al., 2012). In patients suffering from therapy failure, including induction of chemoresistance and radioresistance, distant metastasis before a surgical operation has been discovered (Rossi et al., 2014). Pancreatic cancer is characterized by diverse mutations, including RAS, Smad4, and p53 and thus frequently exhibits chemoresistance (Kim and Tannock, 2005) and insensitivity to radiotherapy (Huang et al., 2011). Our earlier study revealed that pancreatic cancer and cancer stem-like cells derived from pancreatic cancer cells have higher levels of long noncoding RNAs and thus induce chemoresistance (Wang et al., 2017). Even so, we still know little about the regulators of malignant behaviors of pancreatic cancer.

Leucine-rich pentatricopeptide repeat-containing (LRPPRC), also known as LRP130, is a member of the pentatricopeptide repeat protein family and exerts multiple functions involving homeostasis, microtubule alterations, RNA stability, DNA/RNA binding, transcriptional activity in mitochondria, metabolic processes, RNA nuclear export, tumorigenesis, and tumor progression (Ghiso and Lennon, 1994; Tsuchiya et al., 2002; Mili and Piñol-Roma, 2003; Mootha et al., 2003; Michaud et al., 2011). LRPPRC is localized to both the cytoplasm and mitochondria (Mili and Piñol-Roma, 2003). In the mitochondrial matrix, LRPPRC binds to single-stranded RNA and thus posttranscriptionally regulates mitochondrial genes and subsequently regulates mitochondrial functions (Ruzzenente et al., 2012). In cancer progression, LRPPRC was also reported to be associated with mitochondria by interacting with Parkin and thus stabilizing Parkin substrates, including Bcl-2 and Parkin itself to inhibit autophagy, and consequently, LRPPRC protects mitochondria from autophagy degradation (Zou et al., 2013). Knockdown of LRPPRC causes a decrease in Bcl-2, followed by Beclin-1 release to form complexes with PI3KCIII to activate basal levels of autophagy (Zou et al., 2014). In this manner, LRPPRC acts as an autophagy/mitophagy inhibitor *via* maintaining mitochondrial membrane potential (MMP) and thus promoting mitochondrial function (Blackstone, 2015).

Mitochondria play essential roles in physiological processes, including energy production, cell signaling, and apoptosis (Wang and Youle, 2009; Larsson, 2010). Reactive oxygen species (ROS), as a byproduct of energy production in mitochondria, have been shown to promote protein oxidation and consequent misfolding and/or unfolding of mitochondrial proteins localized in the mitochondrial matrix (Niforou et al., 2014; Zorov et al., 2014). Under physiological conditions, the balance between ROS accumulation and ROS scavenging is strictly regulated to avoid oxidative stress, which can regulate the mitochondrial permeability transition pore and thus maintain healthy mitochondrial homeostasis (Zou et al., 2014). By considering that LRPPRC is reported to exert critical roles in maintaining MMP *via* regulating autophagy/mitophagy, it is supposed that LRPPRC might regulate ROS accumulation and scavenge and thus maintain MMP. Previous reports have shown that LRPPRC may act as an oncogene in several kinds of cancer, including hepatoma, lung adenocarcinoma, esophageal squamous cell carcinoma, and colon cancer (Tian et al., 2012); however, the exact role of LRPPRC in pancreatic cancer and whether its regulatory effect on mitochondria is involved in these processes are still unclear.

In this study, we detected the expression level of LRPPRC in 90 pancreatic cancer and paired adjacent tissues and five pancreatic cancer cell lines to investigate the relevance of LRPPRC expression. Furthermore, we also established the potential association of its regulation of mitochondrial function with the malignant behaviors of pancreatic cancer, especially cell proliferation. In conclusion, our results indicated that LRPPRC might be a critical marker for prognosis and a potential therapeutic target in pancreatic cancer.

## Material and Methods

### Clinical Tissue Samples

Our study included 90 patients (57 men, 33 women; mean age 61.9 years; range 36–85 years) recruited from May 2010 and August 2018 after obtaining their written informed consent. All patients who survived from 3 to 7.2 years were confirmed by telephone and mail. The study items included age, sex, tumor size, and tumor–node–metastasis stage. Patient characteristics are summarized in Table 1. Tissues were fixed in 10% formaldehyde, embedded in paraffin, cut into 1.5 mm in diameter and 4 μm in thick, and mounted on a tissue microarray.

**TABLE 1:** Correlation between clinicopathological characteristics and LRPPRC expression.

Total	n	LRPPRC		*p*
		Low	High	
Age				0.361
≤60	40	15	25	
>60	50	20	30	
Gender				0.219
Male	57	21	36	
Female	33	11	22	
Tumor size				0.195
≤5 cm	55	21	34	
>5 cm	35	12	23	
N				0.016^*^
N0	51	21	30	
N1	39	12	27	

* *p*-value for expression levels compared by Mann–Whitney test.

### Immunohistochemical Staining

The tissue microassay was stained for immunohistochemical analysis. Microarray was baked at 60°C for 2 h, deparaffinization with xylene, and then rehydrated after being washed three times in 1× phosphate-buffered saline (PBS). Then, rehydrated microarray was incubated with 3% hydrogen peroxide for 10 min in methanol to inactivate endogenous peroxidase activity and then blocked using 2.5% bovine serum albumin dissolved in PBS against nonspecific binding sites for 30 min at room temperature. Then anti-LRPPRC antibody (diluted in 1:200; Cat. No: ab97505; Abcam, Cambridge, England) was added for overnight incubation at 4°C. Incubated microarray was then rinsed three times in ice-cold PBS and incubated with a horseradish-peroxidase-conjugated antibody (diluted in 1:5,000; Cat. No: ab7090; Abcam) for 1 h at room temperature. The microarray was developed then with 3, 3′-diaminobenzidine solution for 2–5 min, washed briefly in running water, and imaged under a microscope (Olympus BX51; Olympus, Japan).

### Immunohistochemical Analysis

Staining of LRPPRC was mainly detected in the cytoplasm of tumor tissues and slightly observed in the nucleus of tumor tissues. The ratio of positively stained cells, the intensity of stained cells, and staining score were reviewed independently by two pathologists without knowing the clinical features or survival status of the patients. The ratio of positively stained cells was graded as follows: 0 = staining of ≤1%; 1 = staining of 1–20%, 2 = staining of 21–40%, 3 = staining of 41–60%, 4 = staining of 61–80%, and 5 = staining of ≥81%. The intensity of stained cells was graded as follows: 0 = no signal, 1 = week signal, 2 = moderate signal, and 3 = strong signal. The staining score was graded as follows: The ratio of positively stained was graded as follows: low expressing group = the ratio of positively stained cells × staining score ≤ 7.5; high expressing group = the ratio of positively stained cells × staining score > 7.5.

### Cell Culture

The pancreatic cancer cell line Panc-1, SW 1990, MIA PaCa-2, CFPAC-1, and BxPC-3 were incubated in Dulbecco modified Eagle medium (DMEM, Life Technologies, Grand Island, NY, United States) supplemented with 10% fetal bovine serum (FBS, Sigma Chemical Co., St. Louis, MO, United States), penicillin (100 U/ml), and streptomycin (100 U/ml) (Life Technologies, Grand Island, NY, United States) at 37°C incubators with 5% CO_2_. The normal human pancreatic cell line HPC-Y5 was incubated in DMEM and other supplements described earlier. All cells were purchased from the Shanghai Institute of Biochemistry and Cell Biology, Chinese Academy of Sciences (Shanghai, China).

### Cell Viability Assays

Cells were seeded (5 × 10^3^/well) in 96-well plates overnight. After the treatment of doxorubicin (−100 μM) for 24 h, 10-μl tetrazolium salt Cell Counting Kit-8 (Keygen, Nanjing, People's Republic of China) was added to each well (final volume ratio as 10%). Optical density was measured at a wavelength of 450 nm.

### Western Blot

The primary antibodies used was listed as follows: rabbit monoclonal anti-LRPPRC antibody (1:2,000, #ab97505); rabbit monoclonal anti-GFP antibody (1:2,000, #ab290); rabbit monoclonal anti-LC3B antibody (1:1,000, #ab51520); rabbit monoclonal anti-p62 antibody (1:1,000, #ab109012); rabbit monoclonal anti-Bcl-2 antibody (1:1,000, #abab32124); rabbit monoclonal anti-Beclin-1 antibody (1:1,000, #ab208612); rabbit monoclonal anti-PI3KCIII antibody (1:1,000, #ab154598); rabbit monoclonal anti-*β*-actin antibody (1:5,000, #ab8227). Goat anti-rabbit immunoglobulin G H&L antibody (HRP ladled, 1:10,000, #ab7090) was used as secondary antibody. Blot bands were quantified *via* densitometry with ImageJ software (National Institutes of Health Baltimore, MD, United States). *β*-actin was used as an internal reference. To detect the cleavage of LC3-II, LC3-II in Mock + siNC group was considered as 1.

### JC-1 Staining

Cells were briefly washed with PBS three times and incubated with 10 μM of JC-1 (Life Technologies, Grand Island, NY, United States) at 37°C, avoiding light for 15–30 min. The supernatant was removed, and 2 ml PBS containing 5 μg of 4′,6-diamidino-2-phenylindole was added into cultured cells for 5-min incubation at 37°C, avoiding light. Then, cells were rewashed with PBS three times and imaged using a fluorescence microscope (X71, Olympus, Melville, NY, United States).

### Adenosine Triphosphate Detection

Cells were washed with ice-cold PBS and resuspended in detection buffer supplemented with 0.22-M sucrose, 0.12-M mannitol, 40-mM Tricine, pH 7.5, and 1-mM ethylenediaminetetraacetic acid. After 5-min incubation on ice, the sample was analyzed using Optocomp I BG-1 luminometer (GEM Biomedical, Inc.) using the adenosine triphosphate (ATP) Bioluminescent Assay kit (Sigma) following the manufacturer's instruction.

### Real-Time Quantitative Polymerase Chain Reaction

Total RNA was reverse-transcripted into complementary DNA using a reverse transcriptase kit (RIBOBIO, Guangzhou, China). Syber Green Master Mix (Life Technologies) was used and analyzed the relative expressing levels in an ABI7500 system (Applied Biosystems, Foster City, CA, United States) under the following conditions: 95°C 10 min, 60 cycles of 95°C 15 s, and 60°C 1 min. The specific primers used were as follows: LRPPRC, 5′-CTG​CAC​TGT​GCT​CTT​CAA​GC-3′ and 5′-GAC​TGC​ACA​CTA​CCG​AAG​CA-3'; *β*-actin, 5′-AGC​CAT​GTA​CGT​AGC​CAT​CC-3′ and 5′-CTC​TCA​GCT​GTG​GTG​GTG​AA-3'; COX I, 5′-GGA​GCA​GTA​TTC​GCC​ATC​AT-3′ and 5′-CGA​CGA​GGT​ATC​CCT​GCT​AA-3'; COX 3, 5-GAA​CAT​ACC​AAG​GCC​ACC​AC-3′, 5′-TAA​TTC​CTG​TTG​GGG​GTC​AG-3′ and 5'- -3'; ND1, 5′-CTC​CCT​ATT​CGG​AGC​CCT​AC-3′ and 5′-GGA​GCT​CGA​TTT​GTT​TCT​GC-3'; Cyb, 5′-GTC​GGC​GAA​GAA​AAA​TGT​GT-3′ and 5′-AAG​CTG​CTC​ACA​GAG​GGG​TA-3'.

### Staining of Mitochondria

For labeling cells with a mitochondrial marker, 2 ml of DMEM medium was used with 10% FBS containing 100-nM Mitotracker Green/5 µg of 4′,6-diamidino-2-phenylindole per well at 37°C for 30 min. Before imaging, the labeling medium was removed and replaced with a fresh DMEM medium with 10% FBS and imaged with a fluorescence microscope.

### Reactive Oxygen Species Staining

Cells were seeded on six-well plates and cultured with 10-μM 2′,7′-dichlorodihydrofluorescein diacetate (Beyotime, Wuhan, China) for 30 min at 37°C, avoiding darkness. After three washes with ice-cold PBS, cells were imaged using a fluorescence microscope at 488 nm excitation and 525 nm emission wavelengths.

### Cell Cycle Analysis

Cells were suspended and washed with ice-cold PBS to remove the left medium. Cells were fixed with ice-cold 70% ethanol overnight at 4°C. Then, cells were stained with propidium iodide (PI) staining buffer (100 μg/ml RNase A and 40 μg/ml PI in PBS) for 15 min in the dark. Then, cells were analyzed by three laser Navios flow cytometers (Beckman Coulter, Brea, CA, United States).

### Apoptosis Analysis

Cells were suspended and washed with ice-cold PBS to remove the left medium. The cell pellet was resuspended in 1× binding buffer and stained with 5-μl fluorescein isothiocyanate-labeled annexin V at 4°C for 30 min in the dark. Then, 10 μl of PI was added at 4°C for 5 min in the dark. Then, cells were analyzed by flow cytometry using three laser Navios flow cytometers (Beckman Coulter, Brea, CA, United States).

### Migration and Invasion

A total of 2.5 × 10^5^ cells were seeded in a six-well plate and allowed for attaching overnight. The scratch was made with a sterile 10-μl pipette tip. Zero and 24 h later, images were taken.

A total of 5 × 10^3^ cells were seeded into the upper chamber (8-μm pore size; Corning, Inc., Corning, NY, United States) coated with Matrigel (Sigma–Aldrich, St. Louis, MO, United States). Twenty-four hours later, the chamber was fixed with 4% paraformaldehyde and stained with 0.25% crystal violet (Sigma–Aldrich).

### Colony Formation and Tumor Formation

A total of 2 × 10^3^ cells were seeded on six-well plates and maintained in a medium containing FBS for 10–14 days until visible clones appeared. For staining of colonies, 500 μl of Giemsa solution (Keygen, Nanjing, China) was added into each well and incubated for 30 min and removed followed by three washes using PBS.

For performing colony formation in soft agar, each well of a six-well plate that contained 2 ml of 0.5% (w/v) low-melting agar (Sigma–Aldrich, St. Louis, MO, United States) in DMEM medium with 10% FBS was laid in each well. Suspended cells were mixed equally, and 5 × 10^3^ cells in 2 ml of 0.3% low-melting agar in 10% FBS were added above the polymerized base solution. Plates were incubated (37°C, 5% CO_2_) for 14 days before colony number, and diameter was quantified microscopically.

### Real-Time Cellular Analysis

The xCELLigence Real-Time Cellular Analysis system was used to monitor the real-time proliferation. The Real-Time Cellular Analysis Station was maintained at 37°C, 5% CO_2_ incubator 1 h followed by the manufacturer's instruction. For each group, cell viability was analyzed in four replicate wells.

### Statistical Analysis

All statistical analyses were performed using the SPSS version 16.0 software package (SPSS Inc. Chicago, IL, United States). A paired-samples *t*-test was used to analyze the differences between the pancreatic cancer samples and the paired adjacent noncancerous tissue samples. Associations between LRPPRC expression and clinicopathological characteristics were analyzed by the Mann–Whitney test and the Kruskal–Wallis test. Survival curves were estimated using the Kaplan–Meyer method, and the log-rank test was used to calculate differences between the curves. A probability level of 0.05 was chosen for statistical significance.

## Results

### Expression Level of Leucine-Rich Pentatricopeptide Repeat-Containing is Upregulated in Clinical Samples of Pancreatic Cancer and Related Cell Lines

LRPPRC expression was determined by performing immunohistochemistry in 90 pancreatic cancer samples and paired adjacent samples. The number of LRPPRC-positive cells in pancreatic cancer tissues (97.0 ± 9.6%) was significantly higher than that in paired adjacent tissues (57.0 ± 17%, *p* < 0.01). The staining intensity of LRPPRC in pancreatic cancer tissues (1.6 ± 0.3) was significantly higher than that in paired adjacent tissues (1.2 ± 0.2, *p* < 0.05). Consequently, the difference in LRPPRC staining between these paired tissues was statistically significant (*p* < 0.001) (Figures 1A,B). To evaluate the relationship between LRPPRC expression and the prognosis of pancreatic cancer, the Kaplan–Meyer method was used to perform the overall survival analysis. The staining score ≤ 7.5 was considered as low LRPPRC, and >7.5 was considered as high LRPPRC. As illustrated in Figure 1C, the pancreatic cancer patients whose tumors had high levels of LRPPRC had significantly shorter survival than those with no or low levels of LRPPRC (*p* < 0.001). To confirm whether a similar expression pattern of LRPPRC exists in pancreatic cancer cell lines, LRPPRC in pancreatic cancer cell lines, including PANC-1, SW 1990, MIA PaCa-2, CFPAC-1, and BxPC-3, was compared with that in the pancreatic nontumor cell line HPC-Y5. As expected, both the messenger RNA and protein levels of LRPPRC in pancreatic cancer cell lines were significantly higher than those in HPC-Y5 cells (Figures 1D,E). For further *in vitro* experiments, PANC-1 was selected for its high endogenous LRPPRC level.

**FIGURE 1:** Expression of LRPPRC in pancreatic cancer tissues and cell lines **(A)**. Immunohistochemical staining was performed to detect expression levels of LRPPRC in pancreatic cancer tissues compared with adjacent tissues **(B)**. Ratio of positive stained cells (%, *p* < 0.01, *vs*. adjacent tissue, *n* = 90), intensity of stained cells (*p* < 0.01, *vs*. adjacent tissue, *n* = 90), and staining score (*p* < 0.001, *vs*. adjacent tissue, *n* = 90) were presented by scatter plot of LRPPRC expression levels in 90 primary pancreatic cancer tissues **(C)**. Kaplan–Meier postoperative survival curve for patterns with pancreatic cancer and LRPPRC expression was presented to demonstrate correlation between survival time and LRPPRC level in 90 primary pancreatic cancer patients. Messenger RNA **(D)** and protein **(E)** levels of LRPPRC in pancreatic cancer cells were detected and normalized to pancreatic non-tumor cells (*p* < 0.05, *vs*. HPC-Y5).

### Leucine-Rich Pentatricopeptide Repeat-Containing Potentially Inhibits the Basal Level of Autophagy in PANC-1 and BxPC-3 Cells

It was recently reported that in cancer development, LRPPRC associates with mitochondria and thus regulates mitophagy/autophagy (Zou et al., 2014; Zhang et al., 2017), which prompted us to explore whether LRPPRC in pancreatic cancer cells is associated with endogenous cleavage of LC3. Considering that all pancreatic cancer cells present high levels of LRPPRC, PANC-1 and BxPC-3 cells were selected for further experiments after efficient LRPPRC knockdown (Figure 2A). In PANC-1 and BxPC-3 cells, knockdown of LRPPRC obviously increased the number of GFP-LC3 puncta (Figure 2B), and cleaved GFP-LC3-II was also observed to be increased after LRPPRC knockdown (Figure 2C).

**FIGURE 2:** LRPPRC potentially inhibited basal level of autophagy/mitophagy in PANC-1 cells. **(A)** After introduction of short hairpin RNA targets to LRPPRC, protein level of LRPPRC was measured by Western blot to confirm efficient knockdown. **(B)** Localization of cleaved GFP-LC3-I and II were imaged. **(C)** Cleavage of GFP-LC3 was further confirmed by Western blot to detect GFP-LC3-I/II with presence of autophagy inducer, rapamycin. **(D–F)** Western blot was performed to detect expressing levels of endogenous LC3-II and P62 with or without presence of BAF. *p < 0.05, *vs*. Mock group.

Considering that LRPPRC regulates the basal level of autophagy *via* modifying MMP (Zou et al., 2013), we further analyzed the MMP by performing JC-1 staining. As presented in Figure 3A, both LRPPRC knockdown and rapamycin treatment obviously increased the green fluorescence intensity of JC-1 monomers (green), suggesting that knockdown of endogenous LRPPRC has a detrimental effect on MMP, which represents mitochondrial dysfunction. To determine whether endogenous LRPPRC is related to mitochondrial function, reflected by ATP synthesis, mitochondrial DNA copy number, mitochondrial mass, and mitochondrial transcriptional activity, cells after LRPPRC knockdown were used for further analysis. As shown in Figure 3B, knockdown of endogenous LRPPRC significantly decreased ATP synthesis, which was similar to that of the rapamycin-treated group. By detecting mitochondrial gene expression, it was observed that without affecting nuclear gene CDPK3 expression, knockdown of LRPPRC and rapamycin exposure decreased the transcriptional activity of mitochondria (Figure 3C). Further analysis of mitochondrial mass and DNA copy number also showed that knockdown of LRPPRC obviously attenuated the function of mitochondria (Figures 3D,E). To further confirm whether the effects of LRPPRC on mitochondrial homeostasis widely exist in pancreatic cancer cells, we used BxPC-3, which obviously expresses LRPPRC (Figure 1E). Expectedly, knockdonw of LRPPRC presented a detrimental effect on MMP and decreased ATP synthesis, mitochondrial DNA copy number, and mitochondrial transcriptional activity (data not shown).

**FIGURE 3:** Knockdown of LRPPRC-regulated MMP, mitochondrial function, and ROS accumulation. **(A)** After knockdown of LRPPRC and exposure to rapamycin for 24 h, JC-1 staining was performed. JC-1 aggregates (red), monomers (green), and nucleus (blue) were observed to observe mitochondrial homeostasis. After knockdown of LRPPRC and exposure to rapamycin, ATP synthesis was measured, **(B)** transcriptional levels of COX 1, COX 3, ND1, Cyb, and CDPK3 were quantitatively analyzed, **(C)** mitochondrial DNA content was quantitatively analyzed, **(D)** mitochondrial mass was measured by performing mitotracker green staining, **(E)** and ROS accumulation was stained by performing 2′,7′-dichlorodihydrofluorescein diacetate **(F)**, to confirm its effects on mitochondrial function and mass. *p < 0.05, *vs*. shScrambled group; #*p* < 0.05, *vs*. Mock group.

Mitochondrial dysfunction is the main source of ROS accumulation (Zorov et al., 2014). This led us to detect cellular ROS, and the results expectedly showed that knockdown of LRPPRC and exposure to rapamycin obviously increased ROS accumulation (Figure 3F). Taken together, our data indicated that endogenous LRPPRC tightly regulates MMP, mitochondrial function, and mitochondrion-related ROS accumulation.

### Effects of Leucine-Rich Pentatricopeptide Repeat-Containing on Malignant Behaviors in PANC-1 Cells

It is well known that mitochondrial dysfunction regulates the basal level of autophagy/mitophagy and thus regulates the malignant behavior of tumors (Drake et al., 2017). The effects of mitochondrial dysfunction caused by the knockdown of LRPPRC on malignant behaviors in PANC-1 cells are not fully understood. Considering that knockdown of LRPPRC induces ROS accumulation, which is potentially the main cause of mitochondrial dysfunction, the ROS scavenger NAC or MitoQ10 was used after LRPPRC knockdown. As shown in Figure 4A, LRPPRC knockdown significantly inhibited S phase entry of the cell cycle, which was reversed by the addition of both NAC and MitoQ10. Knockdown of LRPPRC failed to affect apoptosis and caspase-9 protein cleavage, which is necessary for mitochondrial-dependent apoptosis, indicating that the regulation of basal autophagy/mitophagy by LRPPRC is not necessary for cell survival without stress (Figures 4B,C).

**FIGURE 4:** Knockdown of LRPPRC regulates malignant behaviors potentially *via* induced ROS. **(A)** To detect effect of LRPPRC on distribution of cell cycle phases, PI staining followed by flow cytometry was measured. **(B)** To detect effect of LRPPRC on cell apoptosis, annexin V-FITC/PI double staining followed by flow cytometry was performed. **(C)** Enzyme-linked immunosorbent assay was performed to measure caspase-9 protein level. **(D)** Scratch assay was performed to detect migrating capacity affected by LRPPRC protein. **(E)** After plating 5,000 or 10,000 cells, a transwell assay was performed to detect invasive capacity affected by LRPPRC. Tumor formation on plats or in soft agar was also measured to present effects of LRPPRC on tumor formation ability **(F,G)**.

Then, we also examined the effects of LRPPRC on malignant behaviors in PANC-1 cells, including migration, invasion, and colony formation. As shown in Figures 4D–G, knockdown of LRPPRC obviously inhibited malignant behaviors, and thus, effect could be reversed by scavenging ROS. Taken together, LRPPRC might regulate malignant behaviors *via* exerting metabolic processes.

### Leucine-Rich Pentatricopeptide Repeat-Containing Desensitizes PANC-1 Cells to Gemcitabine *Via* Inhibiting Reactive Oxygen Species Accumulation Induced by Gemcitabine

Gemcitabine, the main drug of choice for pancreatic cancer patients (Von Hoff et al., 2013; Chiorean et al., 2018), promotes ROS accumulation and thus induces apoptosis, at least in part (Patel et al., 2017). Thus, we examined the effect of LRPPRC on chemosensitivity to gemcitabine. The Cell Counting Kit-8 assay illustrated that knockdown of LRPPRC significantly sensitized PANC-1 cells to gemcitabine, which could be reversed by pretreatment with both NAC and MitoQ10, demonstrating that LRPPRC induced desensitization potentially *via* reducing ROS accumulation (Figure 5A). To examine whether ROS scavengers maintained MMP decreased by knockdown of LRPPRC, JC-1 staining followed by flow cytometry was carried out, and as expected, both NAC and MitoQ10 helped to maintain MMP (Figure 5B). The result of apoptotic induction in response to treatment with 1 μmol/L gemcitabine for 24 h showed that knockdown of LRPPRC increased gemcitabine-induced apoptosis, which was reversed by ROS scavengers (Figure 5C).

**FIGURE 5:** Knockdown of LRPPRC-sensitized PANC-1 cells to gemcitabine *via* promoting ROS accumulation. **(A)** Cell Counting Kit-8 assay was performed to detect gemcitabine sensitivity after LRPPRC knockdown. *p < 0.05, *vs*. shScrambled group; #*p* < 0.05, *vs*. shLRPPRC-1/2 group. **(B)** JC-1 staining was performed, followed by a flow cytometric assay to detect effect of LRPPRC on mitochondrial membrane potential. **(C)** Annexin V-FITC/PI double staining was performed to detect apoptosis after LRPPRC knockdown with or without NAC and MitoQ10 supplement. *p < 0.05, *vs*. shScrambled group; #*p* < 0.05, *vs*. shLRPPRC-1/2 group. **(D)** ROS level was measured after LRPPRC knockdown with or without NAC pretreatment. **(E)** ROS level was measured after LRPPRC knockdown with or without ROS inducers. **(F)** Annexin V-FITC/PI double staining was performed to detect apoptosis with pretreatment of ROS inducers.

To further confirm whether LRPPRC-regulated ROS accumulation is responsible for gemcitabine sensitivity, we first detected that ROS accumulation was obviously promoted after knockdown of LRPPRC and pretreatment with ROSUP or H_2_O_2_ (Figures 5D,E). Notably, LRPPRC knockdown slightly affected ROS level, which indicates its slight effect on endogenous ROS level without gemcitabine treatment. Induction of apoptosis by knockdown of LRPPRC was similar to the effects of ROS accumulation in response to both ROSUP and H_2_O_2_ treatment (Figure 5F). Notably, ROSUP or H_2_O_2_ treatment failed to obviously promote apoptosis in LRPPRC-knockdown PANC-1 cells, indicating that LRPPRC may mainly regulate gemcitabine sensitivity by modifying ROS levels (Figure 5F).

### Leucine-Rich Pentatricopeptide Repeat-Containing Regulates Cell Proliferation Mainly *Via* Inhibiting Mitophagy/Autophagy

Considering that LRPPRC inhibits the basal level of mitophagy/autophagy by interacting with Bcl-2 (Zou et al., 2013) and Beclin-1 (Von Hoff et al., 2013; Zou et al., 2015; Zou et al., 2019), subsequently activating PI3KCIII (Michaud et al., 2011; Ruzzenente et al., 2012), we transiently knocked down LRPPRC, Bcl-2, Beclin-1, and PI3KCIII by transfecting cells with specific small interfering RNAs. In addition, 3-MA, an autophagy inhibitor, was used to inhibit autophagy induced by LRPPRC knockdown. As shown in Figure 6A, knockdown of LRPPRC significantly increased the cleavage of GFP-LC3, which was reversed by the addition of 3-MA, indicating that LRPPRC plays a critical role in inhibiting mitophagy/autophagy. Consistently, LRPPRC was also found to be critical for ATP synthesis *via* inhibiting mitophagy/autophagy (Figure 6B). To determine whether the LRPPRC-modified basal level of mitophagy/autophagy is critical for its regulatory roles in proliferation, cell cycle analysis and real-time cell proliferation assays were performed after LRPPRC knockdown with or without 3-MA addition. As expected, cell cycle blockade in response to LRPPRC knockdown was obviously reversed by the addition of 3-MA (Figure 6C), and the proliferation inhibition in response to LRPPRC knockdown was partially reversed by the addition of 3-MA, indicating that LRPPRC-regulated mitophagy/autophagy is critical for its role as a tumor promoter (Figure 6D).

**FIGURE 6:** Knockdown of LRPPRC inhibited cell proliferation *via* promoting autophagy/mitophagy. **(A)** After knockdown of LRPPRC, Bcl-2, Beclin-1, or PI3KCIII, respectively, protein levels were detected by performing Western blot to determine the potential effects of LRPPRC on regulating LC-3 cleavage. To reveal effects of LRPPRC, Bcl-2, Beclin-1, and PI3K on mitochondrial function, ATP synthesis was detected **(B)** *p < 0.05, *vs*. siScrambled group, cell cycle phases were measured by performing PI staining followed by flow cytometric assay **(C)** real-time cell proliferation assay was performed **(D)**.

## Discussion

Pancreatic cancer is one of the leading causes of cancer-related death worldwide (Siegel et al., 2017). Although the characteristics of pancreatic cancer, such as poor prognosis, late diagnosis, and metastasis, the high rate of chemoresistance is one of the leading reasons for poor prognosis (Storniolo et al., 1999). Gemcitabine is the only first-line chemotherapeutic for pancreatic cancer patients and exhibits only a 12% tumor response rate (Storniolo et al., 1999); the median survival with gemcitabine treatment is still a dismal 5.65 months with a 1-year survival rate of 18% (Lu et al., 2014). In the current study, we used pancreatic cancer cells as a cell model to investigate the molecular mechanism of chemoresistance to gemcitabine. Our results demonstrated that LRPPRC exerted protective effects against gemcitabine in pancreatic cancer cells. LRPPRC dramatically promoted PANC-1 cell survival, proliferation, migration, and invasion and improved mitochondrial function. This study is among the first to report the regulatory roles of LRPPRC in mitochondrial homeostasis and mitochondrial function in human pancreatic cancer cells. Furthermore, we supplied solid evidence to suggest that LRPPRC is upregulated and tightly associated with a low 5-year survival rate. LRPPRC also increased the proportion of cancer cells in G1/G0 cell cycle phases and inhibited cell death (mainly apoptosis). Thus, LRPPRC could be further investigated as a promising target of pancreatic cancer.

LRPPRC tightly regulates the progression of cell cycle phases, probably *via* regulating mitochondrial function and mitophagy. Previous studies have shown that in cancer progression, LRPPRC interacts with Beclin-1 and Bcl-2 and forms a ternary complex to maintain Bcl-2 stability (Zou et al., 2013; Zou et al., 2014), resulting in the maintenance of mitochondrial homeostasis and mitochondrial function. Expectedly, knockdown of LRPPRC causes a decrease in Bcl-2, followed by Beclin-1 release to form complexes with PI3KCIII to activate basal levels of autophagy (Zou et al., 2013). In our study, we found that knockdown of LRPPRC, Bcl-2, Beclin-1, and PI3K or blockage of autophagy with 3-MA decreased autophagy/mitophagy and ATP synthesis. Here, we observed significant promotion of cell proliferation after LRPPRC knockdown, which was reversed by the addition of 3-MA; the regulatory mechanism by which LRPPRC regulates cell proliferation is potentially associated with LRPPRC-regulated autophagy/mitophagy, as suggested by other studies (Li et al., 2014). Accordingly, we hypothesized that LRPPRC might regulate malignant behaviors, including migration, invasion, and chemosensitivity, by regulating mitochondria.

Pancreatic cancer cells, characterized by rapid growth and proliferation, require elevated metabolism, biosynthesis, and energy production (Bhattacharya et al., 2014). Mitochondrial homeostasis and function are essential for physiological processes and energy production. LRPPRC is well known as a regulator of mitochondrial function in cancer progression that acts by interacting with mitochondrial-related proteins, including Beclin-1 and Bcl-2, thus activating PI3KCIII (Zou et al., 2013; Zou et al., 2014). Overexpressed LRPPRC maintains mitochondrial homeostasis by interacting with Beclin-1 and Bcl-2 and maintains MMP (Zou et al., 2013; Zou et al., 2014). In this study, we observed a similar phenomenon in our pancreatic cancer cell line, where LRPPRC expression was relatively high and MMP, mitochondrial ATP synthesis, and malignant behaviors were attenuated by LRPPRC knockdown. Increased autophagy/mitophagy in response to LRPPRC knockdown also inhibited malignant behaviors, which could be reversed by the addition of 3-MA, demonstrating that the regulation of autophagy/mitophagy mediated by LRPPRC is potentially critical.

LRPPRC is a widely expressed protein in human tissues and is deeply involved in metabolic processes. The dysfunction of LRPPRC can cause Leigh syndrome, French–Canadian type, a human disorder characterized by neurodegeneration and cytochrome c oxidative deficiency (Mootha et al., 2003). It was also found to be tightly associated with tumor progression. Vandin et al. (2012) reported that in ovarian cancer patients, mutations in LRPPRC were found to reduce the survival of patients. In prostate cancer, Jiang and colleagues reported that LRPPRC was expressed at a much higher level compared with that in adjacent tissue and positively correlated with tumor grade, metastasis, and serum prostate-specific antigen. These results prompted us to determine whether the expression level of LRPPRC was associated with pancreatic cancer. Expectedly, by performing tissue scanning, it was observed that both the ratio of positively stained cells and the intensity of stained cells in pancreatic cancer tissue presented a higher expression level of LRPPRC in cancer cells compared with that in adjacent tissue, indicating its potential roles in cancer progression. Moreover, a single-cell sequence study, which was considered as a promising technique to evaluate the exact role of LRPPRC in a different subpopulation of interested tissues (Song et al., 2021a; Song et al., 2021b), in further study, is worth performing single-cell sequencing to obtain deep understanding on how LRPPRC affects metabolic processes *via* affecting different subpopulation of pancreatic cancer cells.

## Conclusion

In this study, we show that LRPPRC is highly expressed in pancreatic cancer cells and negatively correlated with survival rate. We also demonstrated that LRPPRC regulated autophagy/mitophagy and maintained mitochondrial function. Consequently, LRPPRC promoted malignant behaviors and chemoresistance in pancreatic cancer cells. Therefore, LRPPRC may act as an oncogene by protecting mitochondria from autophagy/mitophagy-mediated degradation.

## Data Availability

The original contributions presented in the study are included in the article/supplementary material, further inquiries can be directed to the corresponding authors.
